# Performance of Universal Adhesives in Composite Resin Repair

**DOI:** 10.1155/2022/7663490

**Published:** 2022-05-09

**Authors:** Hyemin Yin, Sumin Kwon, Shin Hye Chung, Ryan Jin Young Kim

**Affiliations:** ^1^School of Dentistry, Seoul National University, Seoul, Republic of Korea; ^2^Department of Dental Biomaterials Science, Dental Research Institute, School of Dentistry, Seoul National University, Seoul, Republic of Korea; ^3^Dental Research Institute, School of Dentistry, Seoul National University, Seoul, Republic of Korea

## Abstract

**Aim:**

The objective of this *in vitro* study was to evaluate the bond strength of universal adhesive systems in self-etch and etch-and-rinse modes at the repair interface between aged and new composite resins.

**Materials and Methods:**

Composite resin (Filtek Z250) was thermocycled to represent aged composite resin to be repaired. New composite resin was placed over the aged substrate after surface conditioning: NC (negative control, no surface treatment), A (adhesive only), SBM (Scotchbond Multi-Purpose in etch-and-rinse mode), CSE (Clearfil SE Bond in self-etch mode), SBU (Single Bond Universal), ABU (All Bond Universal), and TBU (Tetric N-Bond Universal). Universal adhesives (SBU, ABU, and TBU) were applied both in etch-and-rinse and self-etch modes. 1 mm × 1 mm × 8 mm beams were sectioned, and microtensile bond strength was measured after 24 hours of water storage and 10,000 thermocycling processes (*n* = 20/group). The fracture surfaces were observed with a scanning electron microscope to evaluate the failure pattern.

**Results:**

The repair bond strength between the old and new composite resins was material-dependent. Universal adhesives significantly improved the repair bond strength (*p* < 0.05), while no significant difference was observed between the etch modes (self-etch or etch-and-rinse) for each universal adhesive (*p* > 0.05). Thermocycling significantly reduced the bond strength in all groups (*p* < 0.05).

**Conclusion:**

Universal adhesives in both etch-and-rinse and self-etch modes outperformed the conventional 3-step etch-and-rinse and 2-step self-etch adhesive systems in terms of resin repair bond strength.

## 1. Introduction

With the advancement of composite restorative materials and adhesive dentistry, composite resin has become a material of choice for direct restorations because the material is economical and esthetic, while requiring minimal cavity preparation [1]. Since all restorations may fail over time due to secondary caries, discoloration, microleakage, and fracture, composite resin could provide another advantage in that the material can be readily repaired rather than being completely replaced. Repair procedures minimize the drawbacks of replacement procedures, which often necessitate a larger cavity preparation and greater expenses [2]. The high resemblance of composite resin to dental hard tissues may cause new resin to be placed over previously placed old resin during the repairing procedure as the complete removal of resin is a very demanding task [3].

In composite resin restorations, adhesive strength is a critical factor associated with the success of the restorations [4]. Commercially available adhesive systems range from 4^th^ generation with a 3-step etch-and-rinse system to a 1-step universal adhesive system [5]. Numerous studies have reported bond strengths between dental hard tissue and composite resin, but there is a lack of studies dealing with the adhesive strength at the interface between aged and fresh resins, which is critical in the repair process. Since the property of aged composite resin has changed because of water absorption and decrease of C=C bonds, it must be treated with a clinically reliable method to maximize the adhesion between aged and fresh resins [6]. The surface condition is also known to be responsible for physical bonding [7]. Sandblasting and silane application are suggested for the repair process of aged resin, but the modification may not be readily performed only at the resin surface without affecting the tooth structure in clinical settings.

Among various types of adhesive systems, universal adhesive has gained popularity with improvements in terms of performance and convenience. In addition, it is the most simplified system that claims to cover the functions of etchant, primer, and adhesive all in a single bottle that could be applied in either etch-and-rinse (total-etch) or self-etch modes. Although there are many universal adhesive products from dental material manufacturers, the composition and concentration of each composition may vary between products [8]. Therefore, the objective of this *in vitro* study was to evaluate the bond strength of universal adhesive systems in self-etch and etch-and-rinse modes at the repair interface between aged and new composite resins. The null hypotheses were that (1) repair bond strength would not be significantly affected by the types of adhesives and that (2) there would be no difference on bond strength between etching modes of universal adhesive systems.

## 2. Material and Methods

### 2.1. Specimen Preparation

A total of 20 composite resin blocks (10 mm × 10 mm × 4 mm) were prepared by placing composite resins (Filtek Z250, 3M ESPE, St. Paul, MN, USA; shade A2 body, lot: N779140) in 3D-printed resin molds (Form 3, Formlabs, Somerville, MA, USA). Two increment layers of 2 mm each were light cured at 1,470 mW/cm^2^ (DeepCure-S, 3M ESPE) for 20 seconds. The last layer was covered with a glass slide in order to obtain a flat surface. The composite-filled blocks were thermocycled at 5°C and 55°C for 10,000 cycles (25-second dwell time) to simulate an aged resin, “old substrate”, to be repaired. Old substrates were wet-grounded with a 320-grit sandpaper corresponding to the approximate roughness obtained by a red-coded fine diamond bur to standardize surface roughness and simulate a clinical condition for composite repair.

The blocks were then randomly allocated into 10 groups according to the surface treatment protocols as follows:

- Group 1: NC: negative control, no treatment
- Group 2: A: adhesive (Scotchbond adhesive, 3M ESPE) was applied and light cured for 10 seconds
- Group 3: SBM in etch-and-rinse mode. Scotchbond Multi-Purpose (3M ESPE) Primer was applied and air-dried for 5 seconds, and adhesive was applied and light cured for 10 seconds
- Group 4: SBU in etch-and-rinse mode. Single Bond Universal adhesive (3M ESPE) was applied for 20 seconds, air-dried for 10 seconds, and light cured for 10 seconds
- Group 5: ABU in etch-and-rinse mode. All Bond Universal adhesive (Bisco) was applied for 20 seconds, air dried for 10 seconds, and light cured for 10 seconds
- Group 6: TBU in etch-and-rinse mode. Tetric N-Bond Universal adhesive (Ivoclar Vivadent) was applied for 20 seconds, air dried for 10 seconds, and light cured for 10 seconds
- Group 7: CSE in self-etch mode. Clearfil SE Bond (Kuraray) Primer was applied for 20 seconds and air dried for 5 seconds, and bond was applied and light cured for 10 seconds
- Group 8: SBU in self-etch mode. Single Bond Universal adhesive (3M ESPE) was applied for 20 seconds, air-dried for 10 seconds, and light cured for 10 seconds
- Group 9: ABU in self-etch mode. All Bond Universal adhesive (Bisco) was applied for 20 seconds, air dried for 10 seconds, and light cured for 10 seconds
- Group 10: TBU in self-etch mode. Tetric N-Bond Universal adhesive (Ivoclar Vivadent) was applied for 20 seconds, air dried for 10 seconds, and light cured for 10 seconds

The name, composition, and manufacturer of each bonding agent used are listed in Table 1, and a schematic outline of the experimental design is shown in Figure 1. The NC (Group 1) served as the negative control in which composite resin was directly placed over the “old substrate” surface without further surface treatment. In A (Group 2), a layer of adhesive was applied on the aged ground substrate prior to composite resin placement. Groups 3-10 were assigned into two major groups by etching mode: etch-and-rinse and self-etch. For the etch-and-rinse mode (Groups 3-6), before applying the adhesive systems, the surface was etched with 37% phosphoric acid (Scotchbond Etchant, 3M ESPE) for 15 seconds and water rinsed and air dried. For the self-etch mode (Groups 7-10), phosphoric acid was not used prior to the application of the adhesive systems. SBM (Group 3) and CSE (Group 7) served as conventional representative adhesive systems for the etch-and-rinse and self-etch adhesive systems, respectively. The three multimode universal adhesive systems were applied in the etch-and-rinse mode (Groups 4-6) and in the self-etch mode (Groups 8-10).

Composite repairs were performed with the same resin composite (Filtek Z250) used for the “old substrate”. New resin layers were applied in 2 increments of 2 mm and light cured for 20 seconds for each layer. The repaired specimens were sectioned into beams (1 mm × 1 mm × 8 mm) under water cooling using a low-speed saw (Mecatome T210, PRESI, Eybens, France) to obtain specimens for microtensile bond strength (*μ*TBS) testing. For each group, the sectioned beams were randomly assigned into the “fresh repair” that were stored in distilled water at 37°C for 24 hours and the “aged repair” that were thermocycled between 5 and 55°C for 10,000 cycles (25-second dwell time) prior to testing (*n* = 20/group).

### 2.2. Measurement of Microtensile Bonding Strength

The 20 sectioned beams for each group were tested using a microtensile tester (Bisco Microtensile Tester; Bisco, Schaumburg, IL, USA). The cross-sectional area (1.0 ± 0.1 mm^2^) was confirmed with a digital caliper. Each specimen was fixed in a custom jig attached to the tester. Tensile load was applied at a crosshead speed of 0.5 mm/min until fracture. The load at failure was recorded in N, and the bond strength was calculated as MPa by dividing the load by the cross-sectional area at the bonded interface. The data obtained were analyzed using one-way analysis of variance and Tukey's honest significant difference post hoc test to evaluate any differences among the surface treatment protocols. The effect of thermocycling on the bond strength of each group was assessed using the independent *t*-test (SPSS Software Version 25, IBM, Armonk, NY, USA), in which an *α* level of 0.05 was employed.

### 2.3. Scanning Electron Microscopy of the Fracture Surface

After *μ*TBS testing, the fractured surfaces of the specimens were mounted on aluminum stubs, sputter coated with gold, and evaluated using a scanning electron microscope (Apreo 2 SEM, Thermo Fisher Scientific) at ×250 and ×1,000 magnification to detect the fracture type-adhesive failure and cohesive failure. Failures that occurred only at the bonding interface were considered adhesive, while those that affected mostly at the substrate or repair composite area were considered cohesive.

## 3. Results

### 3.1. Microtensile Bond Strength

The means and standard deviations of the *μ*TBS measured for all the tested subgroups are presented in Table 2 and Figure 2. In comparison to the negative control group (NC) and adhesive group (A), the *μ*TBS increased significantly in both the etch-and-rinse and self-etch treatment groups (*p* < 0.05). The application of universal adhesive significantly increased *μ*TBS compared to the corresponding conventional adhesive system, regardless of the aging process and etch mode (*p* < 0.05). For both the fresh and aged repair groups, SBU exhibited the highest value (65.90 MPa for fresh repair and 46.29 MPa for aged repair in the etch-and-rinse mode; 62.28 MPa for fresh repair and 51.76 MPa for aged repair in the self-etch mode). All the groups, irrespective of etch mode and surface treatment protocols, demonstrated lower *μ*TBS after aging (*p* < 0.001). Regarding the reduction percentage of *μ*TBS after thermocycling, SBU showed the lowest reduction (16.9%) followed by ABU (20.0%), both in the self-etch mode. The application of adhesive (A) increased *μ*TBS for the fresh repair group compared to the negative control group (NC), but no significant difference was observed between the two groups after aging.

### 3.2. Scanning Electron Microscopy of the Fracture Surface and Failure Mode Analysis

The representative SEM images of adhesive and cohesive failure types are presented in Figure 3.  Figure 4 shows the failure modes among the experiment groups. The dominating failure mode was of the adhesive type regardless of the aging process and etch mode. There was a tendency for increased percentages of cohesive type fractures with higher bond strength. The percentage of cohesive type fractures decreased with the aging process. The SBU group in both the self-etch mode and etch-and-rinse mode, which has the highest bond strength, exhibited the highest number of cohesive failures. The lowest bond strengths for the etch-and-rinse mode and self-etch mode, SBM and CSE, respectively, exhibited the lowest cohesive failures.

## 4. Discussion

The present study demonstrated that the bond strength of universal adhesives for composite resin repair was adhesive-dependent. Although no significant difference was found between etch-and-rinse and self-etch modes within each universal adhesive, the universal adhesive systems exhibited significantly greater bond strengths in composite repair than the corresponding multistep adhesive systems. Therefore, the first null hypothesis that repair bond strength would not be different between types of adhesives was rejected, while the second null hypothesis that there would be no significance difference between etching modes of universal adhesive systems was not rejected.

Previous studies have shown varying adhesive strengths in resin repair according to different surface treatments such as silane application, aluminum oxide air abrasion, phosphoric acid etching, and hydrofluoric acid etching [6, 9–15]. The surface treatment of aged resin serves two purposes: to remove the superficial layer altered by the saliva exposing a clean, higher energy composite surface for wettability, and to increase the surface area through the creation of surface irregularities [11]. In this study, adhesives were applied on the substrates that were wet-grounded with a 320-grit sandpaper to mimic clinical situations where a red-coded diamond bur is used to prepare the tooth and previously placed composite resin for resin repair. Wendler et al. [6] reported increased adhesive strength to aged resin upon phosphoric acid etching because of improved surface energy and surface wettability through the cleansing of surface debris [2]. In the present study, the bond strength of universal adhesives was not clearly affected by phosphoric acid etching procedures, as was also shown by the study from Şişmanoğlu et al. [9] The function of additional phosphoric acid etching may have been compensated by surface preparation by grinding followed by copious water irrigation to remove debris and possible contaminants prior to the surface conditioning procedure. However, the use of phosphoric acid etching could be recommended when the ground composite resin gets contaminated by oral fluids such as saliva and blood.

3-step SBM and 2-step CSE, which are regarded as so-called conventional gold standards for etch-and-rinse and self-etch systems, respectively, exhibited significantly lower repair bond strength than all three kinds of universal adhesive systems. Cakir et al. [13] also demonstrated improved bond strengths of SBU and ABU compared to CSE. The improvement of repair bond strengths of universal adhesives could be explained by the incorporation of 10-MDP, which can create chemical bonding with various surfaces including zirconia fillers incorporated in a composite resin material [16]. However, the mere presence of 10-MDP cannot be a conclusive factor since CSE also contains 10-MDP in the primer. Therefore, it could be speculated that the repair bond strength is influenced by the chemical formulations in each adhesive because not all universal adhesives contain the same concentration or purity of 10-MDP [8]. This suggests that the separate priming and adhesive procedure is not helpful in resin repairs compared to resin bonding to tooth substrate.

Some universal adhesives contain silane coupling agents because surfaces coated with silane are more reactive for repair resin and increase the wettability which improves the infiltration of the bonding agent into the surface microretentions [6, 12, 15, 17]. Silane contains (i) silanol groups, which reacts with exposed inorganic filler particles of the aged composite substrate, and (ii) organofunctional groups, which react and copolymerize with the methacrylate groups of the repair material [18]. Previous studies have reported that the application of silane before adhesive procedures or the use of a silane-incorporated universal adhesive improved the bond strength of aged resin composite [13, 19]. Şişmanoğlu et al. [9] showed that SBU exhibited higher cohesive failure rates and the highest bond strength while maintaining repair *μ*TBS after thermocycling when compared to other universal adhesives. Similarly, in this study, SBU showed the highest repair bonding strength with more cohesive failures in both etch-and-rinse and self-etch modes and the lowest reduction rate in bond strength after aging. Nevertheless, silane in universal adhesives was found to be not as stable long term because of hydrolysis and dehydration condensation facilitated by the low pH of the adhesives [20]. Further investigation is required to evaluate the stability of silane incorporation in universal adhesives. In contrast to our findings, Cuevas-Suarez et al. [14] indicated different consequences that TBU exhibited higher or similar bonding strength to SBU. The difference in the findings between this study and previous related investigations may be explained by the different materials and methodologies employed for bond strength evaluations.

Aging is one of the important factors limiting the longevity of adhesive restorations. The aging process deteriorated bonding strength in all adhesive systems tested in the present study. During the aging process, water molecules penetrate the resin matrix and resin-adhesive interface and cause hydrolysis within the material [21]. In this study, the aging process of composite resin in clinical situations was simulated by thermocycling at 5°C and 55°C for 10,000 cycles. It has been proposed that approximately 10,000 cycles could simulate a service year in oral environment [22]. Thermocycling generates stresses due to differences between the thermal expansions of various materials that could result in bond failure at the tooth-restoration or filler-matrix interface [23]. Rinastiti et al. [24] demonstrated increased surface roughness and lower repair bond strength after aging. In the present study, the thermocycling process led to a significant reduction in bond strength, regardless of the etching mode and type of adhesive. This was confirmed by fracture type analysis where the percentage of cohesive failure decreased after thermocycling, suggesting reduced adhesive strength at the bonded interface.

The limitation of this study was that the type of failures could not be easily distinguished between the repair and substrate due to the same resin and shade used as a repair and substrate material. Only a single methacrylate-based microhybrid composite resin was used to allow for standardization to focus on the variables in the adhesive systems. Various composite resins have different surface characteristics depending on the composition of the filler particles and resin matrix. Altinci et al. [4] tested the repair bond strength of different composite resins with a universal adhesive and presented inconsistent bonding strengths when the same surface treatment was applied on different types of composite resins. The authors suggested that bigger filler particles may provide extra retentive areas after surface roughness treatment, thereby resulting in easier retention of new composite layers [4].

The findings of this study cannot be generalized, but it provides general overviews of the potential effects of universal adhesive in composite resin repairs using either etch-and-rinse or self-etch modes. Within the limitations of the study, the universal adhesive systems significantly improved the repair bond strength between old and new composite resins compared to the conventional multistep adhesive systems. Since no significant difference was observed between etch modes, the clinician should evaluate the surroundings and surface to be repaired before deciding on whether to precondition the surface with phosphoric acid. Considering the reliable bonding capabilities of universal adhesives on both teeth and composite resins, the application of universal adhesives, particularly SBU, could be recommended for composite repairs, especially when the boundary between tooth structure and composite resin cannot be easily discernible.

## 5. Conclusion

The repair bond strength between old and new composite resins was found to be material-dependent. Universal adhesives significantly improved the repair bond strength, while no significant difference was observed between the etch modes (self-etch or etch-and-rinse) for each universal adhesive. Although thermocycling significantly reduced the bond strength in all groups, universal adhesives outperformed the conventional 3-step etch-and-rinse and 2-step self-etch adhesive systems in terms of resin repair bond strength.

## Figures and Tables

**Figure 1:** Experimental design of the study. NC: negative control; A: adhesive; SBM: Scotchbond Multi-Purpose; SBU: Single Bond Universal; ABU: All Bond Universal; TBU: Tetric N-Bond Universal; CSE: Clearfil SE Bond.

**Figure 2:** *μ*TBS of fresh repair (a) and aged repair (b). NC: negative control; A: adhesive; SBM: Scotchbond Multi-Purpose; SBU: Single Bond Universal; ABU: All Bond Universal; TBU: Tetric N-Bond Universal; CSE: Clearfil SE Bond. Different superscript capital letters and lowercase letters were statistically significantly different among fresh and aged repairs, respectively.

**Figure 3:** SEM images of the fracture surface. Adhesive failure: (a) ×250 and (b) ×1,000 magnifications. Cohesive failure (c) ×250 and (d) ×1,000 magnifications.

**Figure 4:** Analysis of fracture type. A: aged repair; F: fresh repair.

**Table 1:** Adhesives used in the study.

Materials (code, lot number)	Manufacturer	Chemical composition
Scotchbond Multi-Purpose (SBM, primer: N998661 and adhesive: N887579)	3M ESPE, St. Paul, MN, USA	Primer: water, HEMA, copolymer of acrylic and itaconic acids Adhesive: HEMA, BISGMA
Clearfil SE Bond (CSE, primer: 640305 and bond: 6J0490)	Kuraray, Osaka, Japan	Primer: MDP, HEMA, hydrophilic dimethacrylates, N,N-diethanol p-toluidine, initiators, water Adhesive: MDP, HEMA, BISGMA, hydrophobic dimethacrylates, silanated colloidal silica, N,N-diethanol p-toluidine, initiators
Single Bond Universal (SBU, 90809A)	3M ESPE, St. Paul, MN, USA	HEMA, BISGMA, 2-propenoic acid, 2-methyl-, reaction products with 1,10-decanediol and phosphorous oxide, ethanol, water, 2-propenoic acid, 2-methyl-, 3-propyl ester, reaction products with vitreous silica, copolymer of acrylic and itaconic acid, camphorquinone, dimethylaminobenzoate, ethyl methacrylate
All Bond Universal (ABU, 2000000059)	Bisco, Schaumburg, IL, USA	BISGMA, ethanol, MDP, HEMA
Tetric N-Bond Universal (TBU, Y46487)	Ivoclar Vivadent, Schaan, Liechtenstein	BISGMA, ethanol, HEMA, phosphonic acid acrylate, urethane dimethacrylate, diphenyl phosphine oxide

Chemical composition listed according to composition/information on ingredients in safety data sheet. HEMA: hydroxyethyl methacrylate; BISGMA: bisphenol A-glycidyl methacrylate; MDP: methacryloyloxydecyl dihydrogen phosphate.

**Table 2:** *μ*TBS values (MPa) and reduction by aging (%).

Surface treatment		Microtensile bond strength		
Etch mode	Group	Fresh repair (MPa)	Aged repair (MPa)	Reduction by aging (%)
N/A	NC	33.70 (5.85)^D^	18.68 (3.46)^e^	44.6^∗^

N/A	A	43.67 (2.82)^C^	18.61 (3.70)^e^	57.4^∗^

Etch-and-rinse	SBM	46.52 (6.00)^C^	27.67 (4.23)^d^	40.5^∗^
	SBU	65.90 (7.04)^A^	46.29 (4.71)^ab^	29.8^∗^
	ABU	61.39 (2.52)^AB^	38.96 (3.02)^bc^	36.5^∗^
	TBU	59.78 (3.06)^AB^	41.35 (4.53)^b^	30.8^∗^

Self-etch	CSE	46.34 (3.93)^C^	32.63 (3.59)^cd^	29.6^∗^
	SBU	62.28 (7.62)^AB^	51.76 (8.91)^a^	16.9^∗^
	ABU	57.71 (9.08)^B^	46.18 (7.23)^ab^	20.0^∗^
	TBU	59.47 (9.05)^AB^	36.46 (8.47)^bc^	38.7^∗^

Standard deviation is shown in parentheses. Within the same column, values with different superscript capital letters and lowercase letters were statistically significantly different among fresh and aged repairs (Tukey HSD, *p* < 0.05). ∗ indicates a significant reduction in bond strength of each group after 10,000 thermocycles (*t*-test, where *p* < 0.05). N/A: not applicable; NC: negative control; SBM: Scotchbond Multi-Purpose; SBU: Single Bond Universal; ABU: All Bond Universal; TBU: Tetric N-Bond Universal; CSE: Clearfil SE Bond.

## Data Availability

Brief relevant data are provided in the manuscript.
